This article has been retracted.

# Expression Levels and Clinical Significance of Serum miR-497, CEA, CA24-2, and HBsAg in Patients with Colorectal Cancer

**DOI:** 10.1155/2022/3541403

**Published:** 2022-08-11

**Authors:** Yan Liu, Jie Chen

**Affiliations:** Department of Pathology, Peking Union Medical College Hospital, Chinese Academy of Medical Sciences & Peking Union Medical College, Beijing 100730, China

## Abstract

The objective of the current study was to look at the levels of blood micro ribonucleic acid- (miR-) 497, carcinoembryonic antigen (CEA), carbohydrate antigen (CA) 24-2, and hepatitis B surface antigen (HBsAg) in patients with colorectal cancer (CRC), as well as the clinical importance of these markers in CRC patients. The serum levels of miR-497, CEA, CA24-2, and HBsAg were compared between 60 patients with CRC (observation group) and another 60 patients with colorectal polyps (control group). The 4 indicators in patients with lymph node metastasis and liver metastasis were compared. The diagnostic effects of 4 detection methods and the combined detection were analyzed, and the influence of 4 indicators on the 5-year cumulative survival rate of patients was discussed. The results showed that the serum levels of miR-497 and HBsAg were lower, and the levels of CEA and CA24-2 were higher in the observation group (*P* < 0.05). The combined detection had the best diagnostic effect, and CEA alone had the best prediction effect. The serum level of miR-497 was significantly lower in patients with lymphatic metastasis, with the significantly higher levels of CEA and CA24-2 (*P* < 0.05). The HBsAg level of patients with liver metastases was greatly lower than that of patients without liver metastases (*P* < 0.05). The 5-year cumulative survival rate of patients with high levels of CEA and CA24-2 was significantly lower than that of patients with low level of CEA. The 5-year cumulative survival rate was lower in patients with low level of HBsAg, but the difference was small. The 5-year cumulative survival rate of patients with elevated serum miR-497 was observably lower. In conclusion, combined detection could diagnose CRC more accurately. Serum miR-497, CEA, and CA24-2 were important in the diagnosis of lymph node metastasis of CRC. HBsAg did a better job of predicting liver metastases in CRC patients. High level of CEA significantly reduced the cumulative survival rate of CRC patients and could predict the long-term survival rate of patients. Serum levels of miR-497, CEA, CA24-2, and HBsAg played a positive role in the diagnosis and evaluation of CRC and could identify lymph node and liver metastases, having a high clinical guidance value.

## 1. Introduction

Colorectal cancer (CRC) is a malignant tumor with high morbidity and mortality, which have been to the second place in western developed countries with more than 1 million deaths per year. In Asia, rectal cancer ranks the third in incidence and has an extremely high mortality among malignant tumors [1, 2]. At present, the early diagnosis rate of CRC is still low, the perception of patients with early symptoms is also low, and the disease gets quite serious generally when it is discovered [3]. The CRC patients are mainly the elderly. With the changes in diet and exercise habits of young people, many young people are accustomed to a high-fat and high-salt diet and have less time to exercise, resulting in decreased digestive function and increased digestive tract diseases. The age range of CRC is also expanding, and many youths also develop CRC, which endangers their life and health [4]. The early detection of CRC patients is difficult, because the early symptoms are not obvious and the patients' attention has not been attracted. After the symptoms become obvious, the disease has developed to a deeper degree, and the treatment will be more difficult. Obvious symptoms begin to emerge after the tumor tissue enlarges. Most patients will have constipation, and some patients will have diarrhea symptoms. The two conditions often alternate, patients may develop intestinal obstruction in the late stage, and some patients will experience anemia and weight loss. Thus, the physical quality of patients has deteriorated sharply, and the difficulty of treatment has increased [5–7]. CRC patients are also prone to tumor cell metastasis, and lymphatic metastasis is relatively common out of tumor metastasis. Surgical treatment for CRC patients with lymphatic metastasis is tough, and it also enhances the tumor treatment complications, such as chemotherapy and radiotherapy which is not helpful to the patients' health recovery. Additionally, liver metastasis is prevalent in CRC patients. When patients with CRC develop liver metastasis, a range of problems develop. This exacerbates the pain hindering the patients' rehabilitation and recovery. Therefore, early diagnosis and early treatment are particularly important in the diagnosis and treatment of CRC.

The most common diagnostic methods for patients with CRC include colonoscopy and serum tumor marker detection [8]. Colonoscopy has a high specificity and sensitivity, allowing it to identify illnesses more precisely; yet, the expense of colonoscopy is high, putting patients under financial strain and reducing their bearing capacity. In addition to it, colonoscopy necessitates a high level of skill and expertise on the part of the doctors. Patients will be harmed if the procedure is performed incorrectly, and the colorectal mucosa at the operation site will be destroyed, producing more agony and pain for the patients. As a result, patients are susceptible to more fear and anxiety, and they are often unwilling to undergo such kind of examination [9–11]. What makes CRC examination approach more reliable, painless, and cost-effective for patients is serum tumor marker examination. Its significance is that it can be repeated and is more convenient to get supplies and material. It offers clear advantages in CRC inspection and diagnosis, as well as more accurate examination results. It has the advantage of possessing high level of acceptability and is applied by both patients and clinicians [12, 13]. Serum tumor markers can detect malignant tumors more accurately, this method is relatively simple to operate, and patients suffer less pain as well as less damage, having a wide range in applications [14, 15]. Common tumor markers include carcinoembryonic antigen (CEA) and carbohydrate antigen (CA) 24-2 [16, 17]. CEA is a structural protein and one of the components of cell membranes; it can be detected in the serum of patients with CRC [18]. Elevated CEA is common in gastrointestinal tumors, urinary tract tumors, lung cancer, breast cancer, and other diseases. However, colitis, pancreatitis, etc., can also increase serum CEA in patients [19, 20]. CEA has an important auxiliary value in diagnosing malignant tumors. CA24-2 is a glycosphingolipid antigen widely used in the diagnosis of malignant tumors, especially tumors of the digestive tracts. It is a common choice for the diagnosis of CRC patients with high sensitivity and specificity. Micro ribonucleic acid- (miR-) 497 is a member of the miR-15 family, closely related to the occurrence and development of various malignant tumors [21]. Hepatitis B surface antigen (HBsAg) is also useful in detecting liver metastases of malignant and cancerous tumors [22]. The HBsAg level of patients with liver metastases is greatly lower than that of patients without liver metastases [23]. The early diagnosis and the judgment of lymph node metastasis or liver metastasis are vital in the diagnosis and treatment evaluation of CRC. In this work, the roles of tumor markers like CEA and CA24-2, miR-497 expression, and HBsAg level were explored and analyzed in the early diagnosis of CRC and lymph node metastasis as well as liver metastasis. The expression of the four-indicator combined detection was also studied in the serum of patients for the early diagnosis of CRC and lymph node metastasis or liver metastasis.

In 60 patients with CRC and 60 patients with colorectal polyps, serum levels of miR-497, CEA, CA24-2, and HBsAg were measured. To diagnose CRC, the clinical effects of the four indications alone and the combination detection were examined and compared. Patients with lymph node metastasis and those without lymph node metastasis were compared using 4 indicators, as were patients with liver metastasis and those without liver metastases. The 5-year cumulative survival rates of patients were also compared between those with high-level and low-level indications. The impact of four indicators on CRC diagnosis and prediction was investigated to give guidance and more possibilities for CRC patient diagnosis. It was also supposed to provide reference for early diagnosis of prediction of lymph node metastasis and liver metastasis.

## 2. Materials and Methods

### 2.1. Research Objects

The objects of this research were 60 patients with CRC and 60 patients with colorectal polyps. The observation group included 60 patients with CRC, and the control group included the other 60 patients with colorectal polyps. The treatment time of the included objects was from January 2013 to December 2015. The mean serum levels of miR-497, CEA, CA24-2, and HBsAg were compared between the two groups. The 4 indicators were also compared of CRC patients with lymph node metastasis and liver metastasis. The 5-year cumulative survival rate was analyzed of patients with positive and negative 4 indicators. The general data of the two groups of patients are displayed in Table 1. This research was carried out with the approval of the ethics committee of the hospital.

Inclusion criteria were listed: (1) The patients were diagnosed with primary colon cancer or rectal cancer. (2) They could offer the complete medical records. (3) They could have the normal communication with nurses. (4) They had no genetic disease. (5) They had no immune disease. (6) They and their families signed the informed consent.

Exclusion criteria were composed of the following: (1) Patients got the secondary CRC caused by metastasis of malignant tumors in other parts. (2) Patients were complicated with metastases to other organs other than liver and lymph nodes. (3) Patients went with heavy psychological burden and difficulty in communication. (4) Patients suffered from other malignant tumors. (5) Patients were complicated with other digestive tract diseases. (6) Patients had severe illness, more complications, and shorter survival time. (7) Patients were unwilling to participate in this research. (8) Patients were unable to participate in the follow-up visits completely.

### 2.2. Methods

#### 2.2.1. Calculation of miR-497 Expression

The cancer tissue mucosa of 60 CRC patients and the colorectal tissue mucosa of 60 patients with colorectal polyps were collected. Samples were taken as soon as possible after isolation, and the total RNA was extracted. The purity and content of the extracted total RNA were identified by a spectrophotometer. Then, the reverse transcription reaction was carried out, the standard samples were prepared, and reverse transcription-polymerase chain reaction (RT-PCR) was conducted. The reaction was determined as specific amplification according to the melting curve. As U6snRNA was taken as the internal reference, the expression of miRNA in the samples was analyzed, and the relative expression level of miR-497 was calculated.

#### 2.2.2. Serum CEA Detection

3 mL of peripheral venous blood was collected from all the objects, centrifuged to separate the serum, which was then stored at -20°C for later use. The CEA in serum was detected by the chemiluminescence method, using an electrochemiluminescence immunoassay analyzer made by the manufacturer F. Hoffmann-La Roche Ltd with the instrument model E-170. When CEA > 5 ng/mL, it was judged to be elevated.

#### 2.2.3. Serum HBsAg Detection

An enzyme-linked immunosorbent test was used to detect HBsAg in the patients' serum. When the S/CO ratio of HBsAg level was equal to or more than 1, it was considered positive.

#### 2.2.4. Serum CA24-2 Detection

The CA24-2 in serum was detected by the chemiluminescence method. The instrument used was an electrochemiluminescence immunoassay analyzer with the model of E-170, produced by F. Hoffmann-La Roche Ltd. When CA24 − 2 > 20 U/mL, it was judged to be elevated. The detection methods of patients' indicators are listed in Figure 1.

### 2.3. Observation Indicators

The disease data of the patients in the observation group were counted, including the depth of infiltration, the degree of tumor differentiation, and the number of cases in different tumor-node-metastasis (TNM) stages.

The expression levels of miR-497, CEA, CA24-2, and HBsAg in serum of patients were determined in the two groups.

The receiver operating characteristic (ROC) curves of the 4 indicators were drawn one by one, and that of the 4-indicator combined detection was also drawn.

The expression levels of miR-497, CEA, CA24-2, and HBsAg in serum were counted of CRC patients with and without lymphatic metastasis.

The expression levels of miR-497, CEA, CA24-2, and HBsAg were also counted in CRC patients with and without liver metastasis.

The line graphs were drawn for the 5-year cumulative survival rate of high-level and low-level CEA, high- and low-level CA24-2, high-level HBsAg and low-level HBsAg, and up- and downregulations of serum miR-497 on CRC patients. CEA was at the low level at 0-15 ng/mL and high at >15 ng/mL. CA24-2 was low at 0-70 U/mL and high at >70 U/mL. HBsAg was at a low level in 0-0.2 *μ*g/L and a high level in >0.2 *μ*g/L. The calculation of the cumulative survival rate was shown as equation (1), where *L* represented the number of surviving cases after *n* months of follow-up, while *Z* represented the total number of cases when the follow-up was started.

(1) $$\begin{array}{c} \text{Cumulative survival rate}=\left(\right)\times 100\%. \end{array}$$

These observation indicators are shown in Figure 2 below.

### 2.4. Statistical Processing

SPSS 20.0 was applied for processing and analyzing the data. The ROC curves of the 4 indicators as well as the combined detection were drawn for the diagnosis of CRC, and *t*-test was for testing. The enumeration data were expressed as rate (%), and *P* < 0.05 was considered to be of statistical significance.

## 3. Results

### 3.1. General Statistics of Patients in Observation Group

Figure 3 displays the general data statistics of the patients in the observation group, in which (a) was of the depth of infiltration, (b) was of the degree of tumor differentiation, and (c) was of the TNM stages. In the observation group, there were 8 patients with the depth of infiltration into the submucosa, 19 cases into the muscular layer, and 33 cases into the serosal layer+subserosal layer. Seven cases got the high tumor differentiation, 28 cases were of moderate differentiation, and 25 cases were of low differentiation. For TNM staging, stage I was found in 13 cases, stage II in 19 cases, stage III in 15 cases, and stage IV in 13 cases. The patients were the most with depth of infiltration into serosal layer+subserosal layer as well as moderate and high differentiation.

### 3.2. Comparison of the Expression Levels of miR-497, CEA, CA24-2, and HBsAg of Patients between the Two Groups

Figure 4 shows the comparison of mean miR-497, CEA, CA24-2, and HBsAg expression levels between the two groups of patients. Figures 4(a)–4(d) represent the mean miR-497, the mean CEA, the mean CA24-2, and the mean HBsAg, respectively. The mean serum miR-497 was 5.29 in the control group and 1.57 in the observation group. The mean CEA of patients in the control group was 10.32 ng/mL, and that in the observation group was 19.27 ng/mL. The mean CA24-2 was 55.67 U/L and 73.92 U/L in the control and observation groups, respectively. The mean HBsAg in the control group and observation group was 0.38 *μ*g/L and 0.22 *μ*g/L, respectively. The mean serum miR-497 and mean HBsAg levels in the observation group were significantly lower than those in the control group. The mean CEA and mean CA24-2 levels were significantly higher than those in the control group. The differences showed the statistical significance (*P* < 0.05).

### 3.3. The ROC Curves of the Separate Detections and Combined Detection of the 4 Indicators in the Diagnosis of CRC

The ROC curves of the 4 indicators and the combined detection are presented in Figure 5 for the diagnosis of CRC. In the diagnosis of CRC, combination detection had the best predictive impact. CEA had a greater prediction impact than the other three approaches, with HBsAg being the poorest.

### 3.4. Correlation of the 4 Indicators and Lymph Node Metastasis of CRC

Figure 6 displays the correlation of 4 indicators and CRC lymph node metastasis, in which Figures 6(a)–6(d) represent mean miR-497, mean CEA, mean CA24-2, and mean HBsAg, respectively. The mean miR-497 level in patients with lymph node metastasis was 1.42, while that in patients without lymph node metastasis was 1.67. The mean CEA level was 20.78 ng/mL and 18.69 ng/mL in patients with and without lymph node metastases, respectively. The mean CA24-2 levels in patients with lymph node metastasis and those without lymph node metastasis were 83.27 U/L and 67.23 U/L, respectively. The mean HBsAg levels in patients with and without lymph node metastases were 0.22 *μ*g/L and 0.21 *μ*g/L, respectively. The mean serum miR-497 level was significantly lower in patients with lymph node metastasis, and the mean CEA and mean CA24-2 levels were significantly increased (*P* < 0.05). There was no significant difference in the mean HBsAg level between the two groups (*P* > 0.05).

### 3.5. Correlation of the 4 Indicators and Liver Metastasis of CRC

In Figure 7, the correlation between the 4 indicators and liver metastases of CRC was analyzed. Figures 7(a)–7(d) show the mean serum miR-497, mean CEA, mean CA24-2, and mean HBsAg levels, respectively. The mean serum miR-497 levels in patients with liver metastases and those without liver metastases were 1.59 and 1.62, respectively. The mean CEA levels in patients with and without liver metastases were 19.77 ng/mL and 19.26 ng/mL, respectively. The mean CA24-2 level was 78.94 U/L in patients with liver metastases and 79.63 U/L in patients without liver metastases. The mean level of HBsAg in patients with liver metastasis was 0.08 *μ*g/L, while that in patients without liver metastasis was 0.36 *μ*g/L. The mean miR-497, mean CEA, and mean CA24-2 levels in patients with liver metastases were not significantly different from those without liver metastases (*P* > 0.05). The mean HBsAg levels were significantly lower in patients with liver metastases (*P* < 0.05).

### 3.6. Influence of 4 Indicators on the Cumulative Survival Rate of CRC Patients

The effect of CEA on the cumulative survival rate of CRC patients is displayed in Figure 8. The 5-year cumulative survival rate of patients with high-level CEA was remarkably lower than that of patients with low-level CEA.  Figure 9 shows the effect of CA24-2 on cumulative survival rate of CRC patients. The 5-year cumulative survival rate of patients with high level of CA24-2 was much lower than that of patients with low level of CA24-2.  Figure 10 represents the effect of HBsAg on cumulative survival rate of CRC patients. The 5-year cumulative survival rate of patients with low level of HBsAg was notably lower than that of patients with high level of HBsAg, but the difference was quite small. The effect of serum miR-497 is presented in Figure 11. The 5-year cumulative survival rate of patients with increased miR-497 was greatly lower than that of patients with decreased miR-497. High-level CEA greatly reduced the cumulative survival rate of CRC patients and was the major predictor of long-term survival rate in CRC patients.

## 4. Discussion

CRC is a common cancer with a high mortality. CRC patients will have a series of gastrointestinal symptoms, which will make the physical condition of patients worse. Many systemic symptoms will emerge in the later stage, bringing pain to the patients and making the treatment more difficult [24]. CRC patients often have lymph node metastasis and liver metastasis, which will aggravate the condition and threaten the life safety of patients. Lymphatic vessels are the main route of metastases for many tumors, and lymph node metastasis is the major cause of death in many patients with malignant tumors [25]. Patients with CRC are prone to regional lymph node metastasis in the early stage. Tumors spread to lymph nodes through lymphatic vessels, making treatment difficult for patients and the high mortality [26]. The liver is also the site where CRC patients are prone to metastases. The treatment of CRC is more difficult after liver metastasis with high risk, and the mortality is greatly increased. The liver metastasis will make the treatment of CRC patients difficult. Patients with liver metastasis from CRC need to undergo surgical treatment, but patients with liver metastasis cannot meet the criteria for surgical resection when the disease is discovered. Furthermore, follow-up conversion therapy is required; after that, a surgery can be performed according to the patients' situation [27, 28]. The early diagnosis is extremely important to the prognosis of CRC patients. Early detection and early treatment are the important ways for the disease control and treatment. Interventions can be given before the disease worsens and spreads to improve the prognosis and increase the survival years of patients with CRC. The accurate judgment of lymph node metastasis and liver metastasis is an important measure to promote CRC patients to receive treatment as soon as possible. Therefore, it is extremely important to explore the evaluation indicators of lymph node metastasis and liver metastasis in patients with CRC, which has become a research hotspot in clinical practice.

The prognosis of CRC patients is generally poor. If it is not discovered and treated timely, lymphatic metastasis and liver metastasis are prone to occurrence. In such a case, the condition of patients will be aggravated, the difficulty for the treatment will be increased, and the mortality will be improved. Early examination and diagnosis can promote the early acceptance of patients to the treatment, improving the prognosis; therefore, it requires a suitable detection method for diagnosing the disease. Common CRC diagnosis methods mainly consist of colonoscopy and serum tumor markers. Although the colonoscopy has a high accuracy, the detection process will bring fear and pain to the patients, and the tolerability and recognition degree of patients are low. Serum tumor biomarkers can be used for early diagnosis of malignant tumors, with less pain in the test. It is easy to accept with the lower cost, having the extensive application at current. CEA and CA24-2 are two serum tumor markers in the diagnosis of CRC. CEA is for tumor screening of CRC with a high sensitivity, and the results are usually more accurate. It shows a high diagnostic value of CRC, but the sensitivity and specificity lack in the general population. The prognosis accuracy of CEA will be affected in patients with CRC complicated with type II diabetes. The CEA level of type II diabetes patients is higher than that of nontype II diabetes patients [29]. In patients with normal initial level of CEA, the postoperative CEA level and variations may be effective markers for evaluating tumor progress; TNM staging combined with CEA levels may be more accurate in the prognostic prediction of CRC patients [30]. CEA, CA24-2, and CA19-9 in serum have the clinical value in CRC detection as well. As the level of tumor markers and gene mutations of KRAS/NRAS/PIK3CA/BRAF are detected, it can be found that the concentrations of CEA, CA24-2, and CA19-9 of patients with CRC are quite higher. The sensitivity of these tumor markers is arranged in the descending order as CEA>CA19-9>CA24-2. The specificity is the best of CA24-2, followed by Ca19-9 and CEA, which were all more than 92% [31]. Dai et al. [32] found that the combination of MIC-1, CEA, CA19-9, and CA24-2 had the highest sensitivity and specificity for CRC diagnosis. miRNA has an inhibitory effect on the translation of target mRNA, influencing the growth, reproduction, and metabolism of cells. It is important in the occurrence and development of tumors. The expression of miR-497 will show a downregulation considerably in a variety of tumors, having a high value in clinical diagnosis. Zou et al. [33] discussed the expression model of serum miR-497 in CRC patients, and the diagnostic value of miR-497 for CRC was verified. The serum miR-497 was found to be the independent prognostic factor of CRC, and it could be used as a biomarker for CRC diagnosis and prognosis. The disordered miRNA will affect the development of cancers strikingly. miR-497 and its target gene B cell lymphoma 2 (BCL2) may be related to the adverse prognosis of cancer patients. The expression ratio of BCL2/miR-497 has a close relationship with disease development in patients with CRC, miR-497 is in relation with clinical pathological characteristics and CRC prognosis, and the expression ratio of BCL2/miR-497 is correlated with poor CRC prognosis and short survival. HBsAg has an important role as well in diagnosing liver metastasis in patients with CRC [34]. Studies have shown that the mortality is higher in the HBsAg-positive male patients with CRC [35]. Therefore, miR-497, CEA, CA24-2, and HBsAg levels in serum are of positive significance in diagnostic and prognostic applications of CRC diseases.

The serum miR-497, CEA, CA24-2, and HBsAg levels were explored on the diagnosis effect of CRC in this work. These 4 indicators were compared of patients with CRC and colorectal polyps, and those were also compared between patients with lymph node metastasis and liver metastasis. The 5-year cumulative survival rates were analyzed under the 4 indicators, and the analysis was also performed for patients with high- and low-level indicators. miR-497 level and HBsAg level were greatly lower, and CEA and CA24-2 levels were dramatically higher in the observation group (*P* < 0.05). From the ROC curves of separate detections and combined detection of 4 indicators, combined detection was more advantageous for diagnosis of CRC; in separate detections, CEA showed the better predictive effect than others. miR-497 level in lymphatic metastasis patients was lower than that in nonlymph metastasis patients significantly, and CEA and CA24-2 levels were higher than those in nonlymph metastasis patients significantly (*P* < 0.05). Thus, miR-497, CEA, and CA24-2 have high values for the prediction and diagnosis of lymph node metastasis of CRC. miR-497, CEA, and CA24-2 levels were not significantly different in liver-metastasis patients from those with no liver metastasis (*P* > 0.05), while HBsAg level was lower than that of patients without liver metastasis remarkably (*P* < 0.05). Thereout, HBsAg was of great role in the prediction of liver metastasis in CRC patients. The 5-year cumulative survival rates of patients with high-level CEA and high-level CA24-2 were considerably lower than those of cases with low-level CEA and low-level CA24-2. The rate for low-level HBsAg patients was relatively low; however, the difference was not significant. The 5-year cumulative survival rate of patients with miR-497 downregulation was highly reduced. From the above, high level of CEA had an effect of significantly reducing the cumulative survival rate of CRC patients and predicting long-term survival rate more accurately. miR-497, CEA, CA24-2, and HBsAg levels in serum were of great significance in the diagnosis and survival prediction of CRC patients, as they could assess lymph node metastasis and liver metastasis and deserved the clinical application positively.

## 5. Conclusions

In this research, the effects of different examination indicators were compared on the diagnosis and prediction of CRC patients. It was shown that miR-497, CEA, CA24-2, and HBsAg levels had a high diagnostic value for colorectal illnesses and metastases. It could predict disease and patient long-term survival and encouraged patients to seek treatment as soon as feasible. miR-497, CEA, and CA24-2 may help with the diagnosis of lymph node metastasis in CRC patients, whereas HBsAg may help with the diagnosis of liver metastasis. Therefore, the 4 indicators had the great clinical application values. Only some of serum tumor markers were selected for detection in this work, and the diagnostic effects of other serum tumor markers as well as indicators were not further explored. In the future, the diagnostic values of other serum tumor markers and detection indicators for CRC could be studied.

## Figures and Tables

**Figure 1:** Detection methods of patient indicators.

**Figure 2:** Observation indicators for the research objects.

**Figure 3:** General statistics of patients in the observation group. (a) The depth of infiltration. (b) The degree of tumor differentiation. (c) TNM stages.

**Figure 4:** Comparison of mean serum expression levels of miR-497, CEA, CA24-2, and HBsAg between the two groups of patients. (a) Mean miR-497. (b) Mean CEA. (c) Mean CA24-2. (d) Mean HBsAg; ^∗^*P* < 0.05 compared to the control group.

**Figure 5:** The ROC curves of the 4 indicators as well as the combined detection in diagnosing CRC.

**Figure 6:** Correlation between the 4 indicators and lymph node metastasis of CRC. (a) Mean miR-497. (b) Mean CEA. (c) Mean CA24-2. (d) Mean HBsAg. ^∗^*P* < 0.05 compared to those without lymph node metastasis.

**Figure 7:** Correlation between the four indicators and CRC liver metastasis. (a) Mean miR-497. (b) Mean CEA. (c) Mean CA24-2. (d) Mean HBsAg. ^∗^*P* < 0.05 compared to those with no liver metastasis.

**Figure 8:** Effect of CEA on cumulative survival rate of CRC patients.

**Figure 9:** Effect of CA24-2 on the cumulative survival rate of CRC patients.

**Figure 10:** Effect of HBsAg on the cumulative survival rate of CRC patients.

**Figure 11:** Effect of miR-497 on cumulative survival rate of CRC patients.

**Table 1:** Comparison of general data of patients in the two groups.

	Gender (male/female)	Age	History of education
Control group	38/22	43.57 ± 8.67	12.32 ± 2.67
Observation group	37/23	42.53 ± 8.33	12.98 ± 2.63

## Data Availability

Data to support the findings of this study is available upon reasonable request from the corresponding author.
